RETRACTED

# Upregulated TRIM29 promotes proliferation and metastasis of nasopharyngeal carcinoma via PTEN/AKT/mTOR signal pathway

**DOI:** 10.18632/oncotarget.7215

**Published:** 2016-02-08

**Authors:** Xiao-Min Zhou, Rui Sun, Dong-Hua Luo, Jian Sun, Mei-Yin Zhang, Meng-He Wang, Yang Yang, Hui-Yun Wang, Shi-Juan Mai

**Affiliations:** ^1^ State Key Laboratory of Oncology in South China, Sun Yat-Sen University Cancer Center, Guangzhou, China; ^2^ Collaborative Innovation Center for Cancer Medicine, Sun Yat-Sen University Cancer Center, Guangzhou, China; ^3^ Department of Nasopharyngeal Carcinoma, Sun Yat-Sen University Cancer Center, Guangzhou, China

**Keywords:** nasopharyngeal carcinoma, TRIM29, metastasis, signal pathway

## Abstract

Tripartite motif–containing 29 (TRIM29) has been reported to be dysregulated in human cancers. Up-regulation of TRIM29 was first observed in NPC cell lines by a genome-wide transcriptome analysis in our previous study. However, its expression biological function and clinical significance in nasopharyngeal carcinoma (NPC) remain unclear. In this study, TRIM29 expression was validated by qRT-PCR and immunohistochemistry in 69 NPC samples. Notably, TRIM29 protein expression was significantly and positively correlated with the tumor size, clinical stage and metastasis. TRIM29 was identified as the direct target of miR-335-5p and miR-15b-5p, both of which were down-regulated and negatively associated with TRIM29 expression in NPC cell lines and clinical samples. Ectopic TRIM29 expression promoted proliferation, epithelial-mesenchymal transition (EMT), migration and invasion in NPC cells, while its depletion inhibited cell invasion and EMT phenotype. Mechanistically, TRIM29 overexpression reduced PTEN expression and increase phosphorylated protein level of AKT, p70S6K and 4E-BP1. Correspondingly, AKT inhibitor and Rapamycin blocked the effect of TRIM29 on cell invasion. In conclusion, our results suggest that miR-335-5p and miR-15b-5p down-regulation results in TRIM29 over-expression, which induces proliferation, EMT and metastasis of NPC through the PTEN/AKT/mTOR signaling pathway.

## INTRODUCTION

Nasopharyngeal carcinoma (NPC) is endemic in Southern China and Southeast Asia, with a high incidence rate of approximately 10-50/100,000 per year [1, 2]. NPC is generally sensitive to radiation therapy and the 5-year survival rate of stage I and II NPC treated with radiotherapy is up to 90% [3]. However, NPC shows the highest metastasis features among head and neck cancers, with 74.5% and 19.9% of patients presenting with regional lymph node metastasis and distant metastasis including bone, liver and lung at the time of diagnosis, respectively [4]. Despite substantial improvements in radiation technique and concurrent-adjuvant chemotherapy during the recent decades, the prognosis for advanced NPC (stage III and IV) is still poor with a 5-year survival rate range from 50% to 70% [5, 6]. Metastasis is the main obstacle in the current clinical management of NPC. Therefore, a clearer understanding of the molecular bases of NPC metastasis is therefore critical for further improving the survival rate of patients with NPC.

RETRACTED

TRIM29 gene, also known as ATDC (ataxia-telangiectasia group D complementing gene), located at chromosome 11q23, was initially identified in a research for the gene responsible for the genetic disorder ataxia-telangiectasia and could increase radioresistance of cells [7]. TRIM29 is a member of the tripartite motif (TRIM) family, which is characterized by a RING finger domain, a B box type 1 (B1) and B box type 2 (B2), and a coiled-coil region [8-10]. Unlike most other TRIM proteins, TRIM29 does not have a RING domain, suggesting that TRIM29 has no E3 ubiquitin ligase activity. The TRIM family of proteins has been implicated in a variety of physiological processes, such as development, oncogenesis, apoptosis and antiviral defense [11-13].

Studies show that TRIM29 has been involved in a variety of cancers. However, the expression levels and biological functions of TRIM29 are different in various types of cancer. Microarray analysis indicates that TRIM29 is over-expressed in lung, pancreatic, gastric, bladder, colorectal, ovarian and endometrial cancers, as well as plasma cell myeloma [14-19]. Moreover, TRIM29 over-expression correlates with poor histological grade, large tumor size, extensive tumor invasion and lymph node metastasis in gastric cancer [20] and invasive phenotype in pancreatic cancers [13], suggesting that TRIM29 functions as an oncogene. Despite its oncogenic effect in certain cancers, TRIM29 is also implicated as a tumor suppressor in some types of breast and bone cancers, and is downregulated in breast and prostate cancers, and cisplatin-resistant oral squamous cell carcinoma cell line [21-25]. These results suggest that the role of TRIM29 might be different, depending on the cell type, its expression level, posttranslational modification and tissue context.

In a previous study, we characterized mRNA and miRNA expression profiles of human NPC cell lines C666-1, CNE2 and non-neoplastic cell line NP69, immortalized from human nasopharyngeal epithelial cells, by RNA sequencing (RNA-seq) (unpublished data). Among the significantly differentially expressed genes, TRIM29 was one of the most highly upregulated genes observed in C666-1 and CNE2 cells compared with NP69 cells (logFC = 9.4 and 10.4, respectively, Supplementary Table 1). TRIM29 mRNA overexpression was further validated in NPC biopsies by using quantitative real-time PCR (qRT-PCR). To the best of our knowledge, TRIM29 expression and its relationship with clinicopathological features in NPC patients have not been characterized yet. Our findings indicate that TRIM29 might play an important role in the development and progression of NPC.

RETRACTED

In the present study, we demonstrate that TRIM29 protein is overexpressed in 69 NPC tissues by immunohistochemistry, and positively correlated with tumor size, clinical stage and distant metastasis. Ectopic expression of TRIM29 in NPC cells promotes cell survival, epithelial mesenchymal transfer (EMT) and invasion/metastasis. Furthermore, our results show that TRIM29 can regulate the key constituent proteins in the PTEN/Akt/mTOR signaling pathway (PTEN, p-Akt, p-p70S6K and p-4E-BP1). Our study suggests that TRIM29, acting as an oncogene, promote EMT, invasiveness and metastasis of NPC cells by activation of the PTEN/AKT/mTOR pathway.

## RESULTS

### TRIM29 is over-expressed and associated with distant metastasis in NPC

With RNA sequencing, TRIM29 mRNA was found to be highly overexpressed in NPC cell lines C666-1 and CNE2 compared with non-NPC NP69 cells, which was confirmed by qRT-PCR. To further verify TRIM29 overexpression in NPC, we employed qRT-PCR to determine TRIM29 expression in 25 snap-frozen NPC tissues and 17 non-cancerous nasopharyngitis (NP) tissues. The result indicates that TRIM29 mRNA expression level is indeed higher in NPCs than in NPs (*p* < 0.05, Figure 1A).

Then we wonder whether TRIM29 protein is also overexpressed in NPC. Western blot analysis was applied to determine protein expression level of TRIM29 in a panel of NPC cell lines (5-8F, 6-10B, S-18, S-26, CNE1, CNE2 and SUNE2). TRIM29 protein is undetectable in non-neoplastic cell line NP69, whereas it can be detected in different expression level in all of NPC cell lines (Figure 1B). Interestingly, the protein expression level of TRIM29 is obviously higher in 5-8F cells with high metastatic potential than in 6-10B cells with low metastatic potential, and also higher in the poorly-differentiated CNE2 cells than in the well-differentiated CNE1 cells, suggesting that TRIM29 may be involved in NPC progression.

To figure out the clinical significance of TRIM29 overexpression in NPC patients, we used immunohistochemistry (IHC) to measure TRIM29 protein expression in 69 NPC tissues. Under a microscope, TRIM29 protein was primarily observed in the cytoplasm of the tumor cells (Figure 1C).

The IHC staining scores for TRIM29 in these NPC samples range from 0.05 to 3, and the NPC samples were classified as high and low TRIM29 expression using the median score (1.88) as the cutoff point. 39 out of the 69 (56.52%) NPC samples were identified as high TRIM29 expressing (staining index > 1.88). The relationship between TRIM29 expression and clinicopathological parameters was analyzed. As shown in Table 1, significant and positive associations were observed between TRIM29 over-expression and tumor size (T1-T2 *versus* T3-T4: 37.5% and 73.0%, *p* = 0.0065), lymphoid metastasis (N0-1 *versus* N2-3: 42.5% and 79.3%, *p* = 0.0049), distant metastasis (M0 *versus* M1: 23.1% and 53.3%, *p* = 0.0193) and clinical stage (stage I-II *versus* stage III-IV: 13.0% and 47.8%, *p* = 0.0102). No significant associations were found between TRIM29 expression and any other clinicopathological features. All of above results suggest that TRIM29 play an oncogenic role in NPC development and progression.

RETRACTED

**Figure 1:** TRIM29 is highly expressed in human NPC **A.** TRIM29 mRNA levels were validated in snap-frozen human NPC (*n* = 25) and non-cancerous nasopharynx tissues (*n* = 17) by using quantitative real-time PCR analysis. TRIM29 expression was significantly higher in NPC than that in NP tissues (*p* < 0.05, independent Student's *t*-test). **B.** protein expression levels of TRIM29 analyzed by Western blot in a panel of NPC cell lines. Note the higher expression is observed in high metastatic cell line 5-8F compared with the low metastatic 6-10B cells. GAPDH is used as a loading control. **C.** TRIM29 immunostaining of representative samples of NPC with or without metastasis. The scale bar indicates 100 μM (upper lane) or 50 μM (lower lane).

**Table 1:** Relationship between TRIM29 expression and clinicopathologic parameters of NPC patients

Characteristics	Number	TRIM29 protein		*P* value
	of cases	Low(*n* = 30)	High(*n* = 39)	
**Age**				
≤ 50years	40	19(47.5%)	21(52.5%)	0.5854
> 50years	29	11(37.9%)	18(62.1%)	
**Gender**				
Male	50	22(44.0%)	28(56.0%)	0.8965
Female	19	8(42.1%)	11(57.9%)	
**EBV DNA copy**				
≤4000	24	10(41.7%)	14(58.3%)	0.9734
>4000	45	20(44.4%)	25(55.6%)	
**EA-IgA**				
<1:10	17	10(58.8%)	7(41.2%)	0.2592
≥1:10	51	20(39.2%)	31(60.8%)	
**VCA-IgA**				
<1:80	15	5(33.3%)	10(66.7%)	0.5474
≥1:80	54	25(46.3%)	29(53.7%)	
**Tumor size**				
T1-T2	32	20(62.5%)	12((37.5%)	0.0065
T3-T4	37	10(27.0%)	27(73.0%)	
**Lymphatic metastasis**				
N0-1	40	23(57.5%)	17(42.5%)	0.0049
N2-3	29	6(20.7%)	23(79.3%)	
**Distant metastasis**				
Yes	30	14(46.7%)	16(53.3%)	0.0193
No	39	30(76.9%)	9(23.1%)	
**Tumor stage**				
I-II	23	20(87.0%)	3(13.0%)	0.0102
III -IV	46	24(52.2%)	22(47.8%)	

### Upregulated TRIM29 is caused by downregulated miR-335-5p and miR-15b-5p in NPC

Studies have demonstrated that microRNA (miRNA) play a critical role in gene post-transcriptional regulation. Therefore, we hypothesize that TRIM29 overexpression in NPC is caused by dysregulation of related miRNAs. In our previous microRNA-sequencing analysis, the expression of miR-335-5p and miR-15b-5p was found to be obviously down-regulated in NPC cell lines CNE2 and C666-1 compared with non-neoplastic NP69 cells (Supplementary Table 2), while TRIM29 was overexpressed in the two NPC cell lines. This finding was further validated in snap-frozen biopsies of NPC (25 cases) and NP tissues (17 cases) using qRT-PCR in the current study (Figure 2A). These results imply that TRIM29 may be a target of miR-335-5p and miR-15b-5p.

RETRACTED

As expected, TRIM29 is predicted as a target of miR-335-5p and miR-15b-5p in TargetScan and miRanda databases because the sequences of both miRNAs are complementary to the sequences (seed sequences) in the 3′UTR of TRIM29 (Figure 2B). We thus tested whether miR-335-5p and miR-15b-5p could target the 3′-UTR of TRIM29 with dual luciferase reporter assay. As shown in Figure 2C, miR-335-5p or miR-15b-5p overexpression markedly decreases the luciferase activity in 5-8F cells co-transfected with miR-335-5p or miR-15b-5p and reporter gene vector containing the wild-type 3′-UTR sequences of TRIM29 (pMIR-wt-TRIM29-3′-UTR), when compare with the negative control (NC) miRNA. To verify the reduced luciferase activity was caused by the two miRNAs binding to the seed sites, the two seed sequences in TRIM29 3′ UTR were mutated simultaneously. When co-transfected with mutated 3′-UTR sequence of TRIM29 (pMIR-mt-TRIM29-3′-UTR) and miR-335-5p or miR-15b-5p into 5-8F cells, luciferase activity was not changed in these cells compared with the cells transfected with control sequence, indicating that the two miRNAs can directly bind to the seed sequences of TRIM29 3′-UTR. Moreover, 5-8F cells co-transfected with a antagomiR-335-5p or antagomiR-15b-5p and wild type 3′-UTR (pMIR-wt-TRIM29-3′-UTR) have a significantly increased luciferase activity compared with the cells co-transfected with a negative control miRNA and wild type 3′-UTR (Figure 2C), indicating that the antagomiRs have inhibited functions of endogenous miR-335-5p and miR-15b-5p. In order to further verify that miR-335-5p and miR-15b-5p can inhibit TRIM29 expression, the expression level of TRIM29 was examined in 5-8F cells with miR-335-5p and/or miR-15b-5p down-regulation or overexpression. Western blot analysis reveals when miR-335-5p and/or miR-15b-5p expression is suppressed, TRIM29 protein is increased. Conversely, TRIM29 protein is markedly downregulated when both miRNAs are simultaneously upregulated in the same cells (Figure 2D). These results demonstrate that TRIM29 is a target for miR-335-5p and miR-15b-5p, and that TRIM29 over-expression is caused by downregulation of miR-335-5p and miR-15b-5p in NPC.

RETRACTED

**Figure 2:** miR-335-5p and miR-15b-5p regulates TRIM29 expression at the post-transcriptional level **A.** miR-335-5p and miR-15b-5p expression levels were validated in snap-frozen human NPC (*n* = 25) and non-cancerous nasopharynx tissues (*n* = 17) by using quantitative real-time PCR analysis. MiR-335-5p and miR-15b-5p expression was significantly reduced in NPC than that in NP tissues (*p* < 0.001, independent Student's *t*-test). **B.** Predicted miR-335-5p and miR-15b-5p target sequences in the 3′UTRs of TRIM29. **C.** Relative luciferase activity of wt or mutant reporter plasmid co-transfected into 5-8F cells with miR-335-5p or miR-15b-5p mimics together with the negative control, or with miR-335-5p or miR-15b-5p inhibitors with the negative control. Cell lysates were obtained after 48h for analysis. Luciferase activity was normalized to that of the control group to obtain relative luciferase activity. “Wt” represents pMIR-wt-TRIM29-3′-UTR wild-type plasmid vector, and “mt” represents pMIR-mt-TRIM29-3′-UTR mutant reporter plasmid vector. Data were means ± SD (*n* = 3). Asterisks indicate values that are significantly different from the NC group (*P < 0.05, **P < 0.01). **D.** Representative immunoblots of TRIM29 protein expression after treatment with miR-335-5p and miR-15b-5p mimics or inhibitors in 5-8F cells.

### Upregulation of TRIM29 enhances oncogenic growth and inhibits cell apoptosis of NPC

To explore the biologic role of increased TRIM29 in the development and progression of NPC, we generated TRIM29-overexpressing cell lines from both S-18 and 6-10B cell lines (Figure 3A). The MTT and colony formation assays show that over-expression of TRIM29 significantly increase the growth rate of both NPC cells compared with that of control cells (Figure 3B and 3C). We further analyzed cell apoptosis by Annexin V/PI staining and flow cytometry, which showed a dramatically decreased apoptosis in 6-10B-TRIM29 and S-18-TRIM29 cells compared with control cells (Figure 3D). All these results suggest that up-regulation of TRIM29 promotes the proliferation and inhibits apoptosis of NPC cells.

**Figure 3:** TRIM29 promotes NPC cell proliferation and tumorigenesis **A.** Western blot analysis of TRIM29 over-expression efficiency in S18-TRIM29 and 6-10B-TRIM29 cells at a protein level. **B.** MTT assay shows that TRIM29 over-expression in NPC cells promotes cell growth in S-18 and 6-10B cells. **C.** Assessment of clonogenic potentials of the TRIM29 over-expressing cells by counting colony numbers. A remarkable increase in colony numbers was observed in the S-18-TRIM29 and 6-10B-TRIM29 cells in comparison with control. Columns represent the mean value of 3 duplicates; bars represent standard deviation. ** indicates a statistical significance in difference between the indicated 2 bar values (*p* < 0.01). **D.** TRIM29 inhibits apoptosis in NPC cells. 6-10B and S-18 cells expressing empty vector or TRIM29 were collected and stained with PI and Annexin V.

RETRACTED

Tumor growth in nude mice was also performed with S-18-TRIM29 cells. The results show that average weight of tumors formed from TRIM29 overexpressing S-18 cells is significantly heavier than that of control tumors (Figure 4A). With immunohistochemical staining, all tumors formed from TRIM29-overexpressing S-18 cells present strong cytoplasmic positivity for TRIM29 antibody, but only weak signals were found in the tumors from vector-expressing S-18 cells (Figure 4B), indicating that TRIM29 overexpression promotes tumor growth.

**Figure 4:** TRIM29 over-expression promotes NPC tumor growth in xenograft nude mice **A.** Left panel shows images of xenograft tumors at the end of study in nude mice that received a subcutaneous injection of S-18 cells over-expressing TRIM29 or carrying a control vector. Right panel shows weights of individual tumors in the two groups. **B.** H&E and IHC staining for TRIM29 in TRIM29-over-expressing and control tumors derived by S-18 (magnification 200 ×).

### TRIM29 promotes migration and invasion of NPC cells

The above results show that TRIM29 expression is more than 5 times higher in 5-8F cells with high metastatic potential than the paired 6-10B cells with low metastatic potential (Figure 1B). Moreover, TRIM29 expression level in tumor cells is significantly higher in metastatic NPC patients than non-metastatic cases (Table 1). These results suggest a role of TRIM29 expression in NPC metastasis and progression. We hence interrogated the effect of TRIM29 over-expression on NPC cell migration and invasion by both *in vitro* and *in vivo* assays. S18 and 6-10B cells stably expressing TRIM29 were used in wound-healing and transwell migration assays. In wound healing assay, cell migration rate was remarkably increased in TRIM29-expressiong cells as compared with control cells (Figure 5A). In the matrigel coated transwell assay, the average number of the migrated cells in TRIM29-expressing S-18 group (318 ± 17.09) and 6-10B group (1973.33 ± 64.29) was also significantly higher than that in the control S-18 group (74.67±4.51) and 6-10B group (465.33±13.61), respectively (both *p* < 0.05, Figure 5B).

RETRACTED

**Figure 5:** TRIM29 induces NPC cell migration and invasion **A.** Wound-healing assays show that S18-TRIM29 and 6-10B-TRIM29 cells had higher motility compared with that in control cells. Left, representative images taken at 0 hr and 24 hr after scratching. Right, quantification of cell migration results that are expressed as the mean ± SD of three independent experiments. **p < 0.01 by Student's *t* test. **B.** Cell invasion was evaluated using a matrigel invasion chamber. TRIM29 over-expression increased S-18 and 6-10B cell invasive capacity. Left, representative images of cells that migrated through the PET membrane (magnification 200 x). Right, quantification of cell invasion data. Results are expressed as mean ± SD of three independent experiments. ***p < 0.001 by Student's *t* test. **C.** Knockdown of endogenous expression of TRIM29 in 5-8F cells *via* siRNA transfection was confirmed by Western blot. D. Inhibition of TRIM29 expression leads to much reduced cell invasiveness in 5-8F cells.

To further investigate whether endogenous TRIM29 promotes invasion of NPC cells, loss-of-function studie (siRNA against TRIM29) was conducted. As shown in Figure 5C, endogenous TRIM29 in 5-8F cell was silenced by each of three specific siRNA oligos against TRIM29. Matrigel coated transwell assay was performed in 5-8F cells, which showed that the average number of the invaded cells was 262.67±14.19, 258.33±7.64 and 276.67±3.51, in 5-8F cells transfected with the three different siRNAs, respectively, which were significantly lower than that (1060±121.66) in cells treated with control siRNA (*p* < 0.05) (Figure 5D).

### TRIM29 induces epithelial-mesenchymal transition (EMT) phenotype *in vitro* and promotes metastasis *in vivo* in NPC

The results show that TRIM29 promotes migration and invasion of NPC cell, which suggest that epithelial-mesenchymal transition (EMT) should be involved in these processes. To this end, we used western blot analysis to detect EMT phenotype of NPC cells with TRIM29 over-expression. In TRIM29 over-expressed S-18 and 6-10B cells, the expression of epithelial markers α-catenin and E-cadherin decreased, whereas the expression of mesenchymal markers fibronectin and vimentin were elevated compared with the control cells (Figure 6A). The opposite results were obtained from the 5-8F cells transfected with specific siRNAs against TRIM29 (Figure 6B). Taken together, these data strongly suggest that TRIM29 over-expression can induce EMT in NPC cells.

**Figure 6:** TRIM29 expression promotes NPC cell epithelial-mesenchymal transition and metastasis in nude mice **A.** Western blotting reveals a reduced expression of epithelial makers (E-cadherin and α-catenin) and an increased expression of mesenchymal markers (fibronectin and vimentin) in TRIM29-expressing S-18 and 6-10B cells in comparison with the vector controls. GAPDH was used as a loading control. **B.** Western blotting assay shows increased levels of E-cadherin and α-catenin, and decreased levels of fibronectin and vimentin in 5-8F-shTRIM29 cells compared with that in shNC treated cells. **C.** Over-expression of TRIM29 promoted S-18 cell invasion and metastasis in athymic nude mice *in vivo*. Left, representative images show lungs with metastatic NPC tumors; left (lower), number of metastatic nodules formed in the lung of mice 6 weeks after tail vein injection of S-18-vector and S-18-TRIM29 cells (5 mice per group; *p* < 0.01; independent Student's *t-*test); right, Examples of haematoxylin and eosin staining in two lung samples originating from S-18-vector and S-18-TRIM29 cell-injected mice (magnification 400×).

RETRACTED

The *in vitro* experiments above show that TRIM29 promotes migration, invasion and EMT, all of which can facilitate metastasis of NPC cells. To confirm that TRIM29 was critical in NPC metastasis *in vivo*, S-18 cells stably expressing TRIM29 or a control sequence were injected into the tail vein of nude mice. Eight weeks after injection, the mice were sacrificed, and metastatic tumor nodules formed in the lung were examined. A much greater number of metastatic nodules are found on the surface of the lung in mice treated with TRIM29-overexpressing NPC cells than those with the control cells (Figure 6C). These observations indicate that TRIM29 overexpression promotes NPC metastasis *in vivo*.

### TRIM29 promotes metastasis in NPC by stimulating PI3K/AKT/mTOR signaling pathway

Since the PI3K/Akt pathway regulates metastasis and is frequently activated in cancer tissues including NPC, we examined the correlation between TRIM29 and the key moleculars of AKT signaling pathway (AKT, P70S6K and 4EBP1) using immunoblotting studies. An increase in the levels of phosphorylated (active) AKT, P70S6K and 4EBP1, but not the total amounts of these proteins, was observed in S-18 and 6-10B cells over-expressing TRIM29 (Figure 7A). Conversely, siRNA-mediated depletion of TRIM29 in 5-8F cells increased the levels of phosphorylated AKT, P70S6K and 4EBP1 (Figure 7B).

**Figure 7:** TRIM29 activates PTEN/AKT/mTOR signal pathway in NPC cells **A.** & **B.** Western blotting analysis reveals that TRIM29 over-expression decreases PTEN and increases phosphorylated protein level of AKT, S6K and 4E-BP1 (pAKT, p-p70S6k and p4E-BP1) expression in S-18 and 6-10B cells (A), whereas knockdown of TRIM29 increases PTEN and decreases the protein levels of pAKT, p70S6k and p4E-BP1 in 5-8F cells (B), without significant changes in total p70S6K, 4E-BP1 and AKT expression. GAPDH was used as a loading control. **C.** Correlation between of TRIM29 and PTEN and p4E-BP1 expression in NPC tissues (*n* = 21). Immunohistochemical staining of representative NPC samples without (left panel) or with metastasis (right panel) (magnification 400×). Pearson correlation coefficient was calculated on the basis of the relative protein expression levels (IHC scores) of TRIM29, PTEN and p4E-BP1 in NPC samples.

RETRACTED

It is well known that the tumor suppressor PTEN negatively regulates the PI3K/Akt pathway [26-28]. Therefore, we compared PTEN expression levels among TRIM29-expressing, siTRIM29-expressing, and control cells. Western blotting results revealed that TRIM29 over-expression led to down-regulation of PTEN protein levels, while TRIM29 silence resulted in a significant up-regulation of PTEN (Figure 7A and 7B), suggesting that TRIM29 negatively regulates PTEN expression.

To explore the clinical relevance of TRIM29 regulation of PTEN/AKT/mTOR pathway in NPC, we performed IHC analysis in 21 NPC tissues, and calculated the correlation coefficients between the expression levels of TRIM29 and the PTEN and p-4E-BP1. We found significant linear correlations between TRIM29 and PTEN (R square = 0.289, *P* = 0.0387), and TRIM29 and p-4E-BP1 (R square = 0.5761, *P* = 0.001) in NPC tissues (Figure 7C). These results support our finding that TRIM29 is involved in PTEN/AKT/mTOR pathway regulation in NPC progression.

To further clarify the importance of PTEN/AKT/mTOR signalling pathway in NPC metastasis, we examined the effects of the AKT inhibitor, mTOR inhibitor rapamycin and siRNA targeting PTEN on the invasion induced by TRIM29. The enhanced invasion in S-18 and 6-10B cells caused by overexpressing TRIM29 was suppressed by treatment of rapamycin (20 ng/ml) (Figure 8A) and AKT inhibitor VIII (20 μM) (Figure 8B). In addition, the reduced invasion of 5-8F cells by TRIM29 inhibition was restored by suppression of PTEN expression by siRNA (Figure 8C). Moreover, suppression of PTEN in TRIM29-repressed cells rescued AKT/mTOR activities of NPC cells (Figure 8D). All of these findings confirmed that the TRIM29 promotion of invasion of NPC cells depends on PTEN/AKT/mTOR signaling.

**Figure 8:** Inhibitors of the PTEN/AKT/mTOR pathway could abolish the effect of TRIM29 on the NPC cell invasion **A.** Invasive abilities of S-18 and 6-10B cells expressing TRIM29 or the empty vector evaluated by Transwell assay after treatment with or without 20 ng/ml of rapamycin. **B.** Invasive abilities of S-18 and 6-10B cells expressing TRIM29 or the empty vector as evaluated by Transwell assay after pretreatment with 20 μM of AKT inhibitor VIII. **C.** Suppression of PTEN expression by siRNA restored the reduced invasion in TRIM29-suppressing 5-8F cells. Transwell assay was performed in 5-8F cells transfected with siRNA-TRIM29, siRNA-TRIM29 plus siRNA-PTEN, or NC. **D.** Suppression of PTEN expression by siRNA in TRIM29-repressed cells rescued AKT/mTOR activities.

RETRACTED

## DISCUSSION

Although the exact functions have yet to be specified, TRIM29 has been shown to increase aggressiveness of certain cancers. It was reported that TRIM29 expression was correlated with poor histological grade, large tumor size, great extent of tumor invasion and lymph node metastasis in gastric cancer [20], and was increasing during the progress from normal pancreatic ductal epithelium to infiltrating cancer, which suggests that up-regulation of TRIM29 promote the development of invasive pancreatic cancer [13]. However, under-expression of TRIM29 in breast and prostate cancer has also been reported using serial analysis of gene expression (SAGE) and DNA microarray analysis [22, 25]. TRIM29 can cause reversion of a malignant phenotype in osteosarcoma and breast cancer cell lines [29]. These reports indicate that the expression pattern and biological function of TRIM29 in carcinogenesis and cancer cell progression may vary depending upon the tissue origin of the neoplasm.

In our previous study with aim to characterize aberrant transcript expression that contribute to the NPC oncogenesis, a combined deep sequencing of human microRNA and mRNA (RNASeq) was used to investigate the expression profiles of NPC cell lines CNE2 and C666-1 and an immortalized nasopharyngeal epithelial cell line NP69 using Illumina Hiseq 2500 (unpublished). There were 1323 and 1106 differentially expressed mRNAs (*p* < 0.05) in C666-1 and CNE2 cells when compared with NP69 cells, respectively. One of the most highly up-regulated genes was the TRIM29 gene, which showed dramatically elevated expression in C666-1 and CNE2 compared with NP69 (logFC = 9.4 and 10.4, respectively) (Supplementary Table 1). Until now, there have not been any studies on the expression and role of TRIM29 in NPC. Subsequently, we confirmed the over-expression of TRIM29 in NPC samples and its positive correlation with tumor size, clinical stage and metastasis of patients. These findings were generally consistent with previous studies that suggested a possible oncogenic function of TRIM29 in certain types of cancers.

The mechanisms by which TRIM29 levels are upregulated in tumors remain unclear. Our microRNA sequencing results show that 169 and 154 microRNAs are differentially expressed in C666-1 and CNE2 against NP69 respectively (*p* < 0.05). Among the deregulated microRNAs, miR-335-5p and miR-15b-5p expression was found to be significantly down-regulated in CNE2 and C666-1 compared with NP69. This result was validated in NPC samples by using qRT-PCR method. Moreover, the bioinformatic method and luciferase reporter assay demonstrate that TRIM29 was a validated target of miR-335-5p and miR-15b-5p, and knockdown of endogenous miR-335-5p and miR-15b-5p increased protein expression of TRIM29 in NPC cells. These results reveal that reduced expression of miR-335-5p and miR-15b-5p result in over-expression of TRIM29 in NPC. Other mechanisms might also be involved in the upregulation of TRIM29 in NPC. Recent studies showed that TRIM29 promoter was hypo-methylated in normal breast epithelium and heavily methylated in other normal epithelial tissues including colon, lung and uterine, and TRIM29 expression inversely correlated with the promoter methylation and was higher in normal breast organoids than in the other tissues [30, 31]. The detailed analysis on NPC specific methylation patterns at TRIM29 promoter needs to be further explored in the future studies.

RETRACTED

Supporting the finding of TRIM29 protein over-expression in metastatic NPC samples, the tumor promoting effects of TRIM29 were also demonstrated by *in vitro* and *in vivo* experiments. In terms of its cellular effects, TRIM29 promoted cell proliferation, colony formation, migration and invasion, EMT, tumor formation and lung metastasis in NPC cells. Reversely, knockdown of endogenous TRIM29 reduced cell migration ability in highly aggressive 5-8F NPC cells. Our findings are in agreement with the previous observation in other cancers that TRIM29 expression increased tumor aggressiveness.

Although the involvement of TRIM29 in carcinogenesis has not been fully elucidated, several recent reports have shown the role of TRIM29 in tumorigenesis examined on the basis of functional studies. Over-expression of TRIM29 promotes the degradation of TIP60 and reduces acetylation of p53 at K120 by TIP60, resulting in an enhancement of cell proliferation and transforming activity [30]. In addition, TRIM29 suppresses apoptosis induced by UV irradiation in HCT116 cell lines through the inhibition of the acetylation of p53 [32]. Evidence from *in vitro* studies indicates that TRIM29 might stabilize disheveled 2, which negatively regulates GSK3β activity in the WNT-β-catenin signalling pathway, resulting in high expression levels of β-catenin in pancreatic cancers [13]. A recent report showed that TRIM29 could promote lung cancer proliferation and up-regulation of cyclin D1 and c-Myc through activation of NF-kB pathway [33].

RETRACTED

To reveal the potential mechanisms underlying the aggressiveness promoting role of TRIM29 in NPC cells, the effect of TRIM29 expression on Akt/mTOR signal pathway were explored. It was reported that activated Akt/mTOR signaling pathway plays a central role in regulating cell proliferation, metastasis, and prevents apoptosis [34]. Activation of Akt is negatively regulated by a well-studied tumor suppressor phosphatase and tensin homolog deleted on chromosome 10 (PTEN) [35-37]. PTEN is thought to suppress tumor cell growth by antagonizing protein tyrosine kinases and regulate the first step of tumor cell invasion and through its interaction with focal adhesions [38, 39]. A disruption of normal PTEN/Akt signaling frequently occurs in NPC, and is correlated with a poor prognosis in NPC [40-42]. PTEN was significantly down-regulated in NPC [28, 42], while the mutation or deletion PTEN was not frequently observed in NPC [43-45], suggesting other mechanisms in NPC are likely responsible for the downregulation of PTEN. In the present study, we identified that PTEN expression was reduced, while the activated proteins in the Akt/mTOR pathway, including p-Akt, p-70S6, and p-4E-BP1 were increased in TRIM29 over-expression NPC cells. The opposite results were obtained when endogenous TRIM29 expression was knockdown by siRNAs in NPC cells. Further correlation analysis in NPC clinical samples showed that TRIM29 expression was positively associated with p-4E-BP1 and negatively associated with PTEN by using IHC analysis. Moreover, inhibitors targeting the AKT and mTOR pathway, and siRNA against PTEN abolished the effects of TRIM29 on cell invasion ability. Collectively, these findings uncover a novel molecular mechanism of activation of PTEN/AKT/mTOR signalling pathway by TRIM29 over-expression and may prove clinical useful in NPC therapy.

Our results proposed that increased expression of TRIM29 in human NPC may be important in the acquisition of an invasive and/or metastatic phenotype, thus favoring the progression of NPC to a more advanced clinic-pathologic stage. The antitumor and radiosensitizing effects of the Akt/mTOR inhibitors have been confirmed in several preclinical studies, which suggest the combination of IR with Akt/mTOR inhibitor might be a promising therapeutic strategy for NPC [46-48]. In the present study, our results showed that AKT Inhibitors and rapamycin abrogate cell invasion ability induced by TRIM29, which indicate inhibitors targeting the Akt/mTOR pathway may be potential for therapy of metastatic NPC expressing high levels of TRIM29. Thus, we propose that TRIM29 might be potentially used as a surrogate biomarker to guide personalized, Akt/mTOR inhibitors-targeted NPC therapy.

RETRACTED

## MATERIALS AND METHODS

### Cell lines and cell cultures

The human NPC cell lines 5-8F, 6-10B, S-18, S-26, CNE1, CNE2 and SUNE2 were maintained in DMEM medium supplemented with 10% fetal bovine serum (Invitrogen, Carlsbad, CA). 5-8F (high tumorigenic and metastatic) and 6-10B (low tumorigenic and metastatic) are subclones of SUNE1. The human immortalized nasopharyngeal epithelial cell line, NP69, was grown in defined-KSFM medium supplemented with EGF (Invitrogen, Carlsbad, CA). All cell lines were cultured at 37°C in a humidified atmosphere of 5% CO_2_.

### Patients and samples

25 cases of fresh NPC tissues and 17 non-cancerous nasopharyngitis (NP) tissues were snap-frozen and stored in liquid nitrogen until further use for qRT-PCR assay. Formalin-fixed, paraffin-embedded tissues (FFPTs) of 69 primary NPC tissues were acquired from the archives of the Department of Pathology in the Cancer center, Sun Yat-Sen University (SYSUCC) between January 2007 and December 2008. Of the 69 NPC patients, 50 were male and 19 were female, with a median age of 50 years (ranged from 37 to 75 years). Clinical information of the samples is summarized in Table 1. The patients were histologically and clinically diagnosed as NPC, assessed according to the TNM staging of International Union against Cancer. None of the patients was subjected to radiotherapy or chemotherapy before biopsy sampling. This study was approved by the Research Ethics Committee of SYSUCC, and written informed consent was obtained from all patients.

### Vectors and transfection

The coding sequences of TRIM29 were amplified and cloned into pEZ-Lv105, an HIV-based lentiviral expression plasmid, and then co-transfected into 293 FT cells with the Lenti-Pac HIV Expression Packaging Kit to generate a recombinant lentiviral particles in accordance with the manufacturers instructions (GeneCopoeia). S18 and 6-10B cells were infected with recombinant lentivirus-transducing units plus 8 mg/ml Polybrene (Sigma, St Louis, Missouri, USA). Stable cell lines expressing TRIM29 were selected using 4 μg/mL puromycin.

Small interfering RNA (siRNA) duplexes specific for TRIM29 and PTEN were purchased from RiboBio Co., Ltd (Guangzhou, China). The negative control RNA duplex (NC) for siRNA was not homologous to any human genome sequence. siRNA or NC at a final concentration of 15nM was transfected into cells in 6-well plates using Lipofectamine 2000 (Invitrogen, CA, USA) according to the manufacturer's instructions. The efficiency of transfection was measured by western blotting 48 h post-transfection.

MiR-335-5p and miR-15b-5p mimics and inhibitors were synthesized by Ribo (Guangzhou, China), respectively. Oligonucleotide transfection was performed with Lipofectamine 2000 reagent (Invitrogen).

RETRACTED

### Quantitative real-time RT-PCR (qRT-PCR)

Total RNA was extracted with TRIzol reagent in accordance with the manufacturer's instructions (Invitrogen, CA, USA). cDNA was synthesised with the PrimeScript RT reagent Kit (Promega, Madison, WI, USA). Real-time PCR was carried out in a total volume of 10 μl, including 8 μl of TaqMan Power SYBR Green PCR Mix (Invitrogen), 0.5 μl of each primer at 25 μM, and 1 μl of cDNA. The quantitative RT-PCR was carried out on the Roche LightCycler^®^ 96 (LC96) real-time PCR platform using the 2^−ΔΔCT^ method. Gene expression results were normalized by internal control GAPDH. Each sample was tested in triplicate.

### Western blot analysis and immunohistochemisty (IHC)

Total proteins were extracted from cultured cells using RIPA buffer containing PMSF and quantified using BCA protein assay kit (Beyotime, Haimen, China). Protein lysates were subjected to SDS-PAGE and transferred onto polyvinylidenedifluoride (PVDF) membrane (Millipore, Billerica, MA) followed by incubating with a primary antibody, and then a secondary antibody. The signals were detected with KeyGEN Enhanced ECL detection kit according to the manufacturer's instructions (KeyGEN, NanJing, China). Rabbit polyclonal antibody against human TRIM29 was purchased from Abcam; mouse monoclonal antibodies against human α-catenin, E-cadherin, fibronectin and vimentin were purchased from BD Biosciences; rabbit monoclonal antibodies against human phospho-AKT (Ser473), AKT (pan), phospho-p70S6K (Thr389), p70S6K, phospho-4E-BP1, 4E-BP1 and PTEN were obtained from Cell Signaling Technology.

Immunohistochemistry (IHC) was performed on 69 cases of formalin-fixed, paraffin-embedded primary NPC tissues. IHC study was performed using a standard streptavidin-biotin-peroxidase complex method. In brief, slides with paraffin sections were deparaffinized and rehydrated. Endogenous peroxidase activity was blocked with 0.3% hydrogen peroxide for 15 min. For antigen retrieval, slides were microwave-treated and boiled in a 10mM citrate buffer (pH 6.0) for 10 min. The slides were incubated overnight at 4°C with rabbit antibody anti-human TRIM29, PTEN, or p4E-BP1, respectively. The staining results were evaluated and scored independently by two pathologists. The intensities were graded as 0 (negative), 1 (weakly positive), 2 (moderately positive), and 3 (strongly positive). The abundance of positive cells was graded from 0 to 100%. The staining score was determined using the following formula: overall scores = percentage score × intensity score.

RETRACTED

### Cell viability assay

Cell viability was measured by a 3-(4, 5-dimethylthiazol-2-yl)-2, 5-diphenyl tetrazolium bromide (MTT) assay (Sigma, St, Louis, Missouri, USA). In brief, cells were seeded in 96-well plates at a density of 1×10^3^ cells/well for 24 h before use. 20μl of MTT solution (5 mg/ml) was added to each well. After a further 4 h incubation, the culture medium was removed and the purple crystals were re-suspended in 150 μl of dimethyl sulfoxide (Sigma). The OD value was measured at 550 nm with a 655 nm reference filter by microplate reader (Bio-Rad, Hercules, CA). Growth rate was calculated as the ratio of the absorbance of the experimental well to that of a blank well. All experiments were performed in triplicates.

### Colony formation assay

S18-TRIM29 and 6-10B-TRIM29 cells and their control cells were placed in six-well plate (300 cells/well) and cultured for 2 weeks. Colonies were fixed with methanol and stained with 0.1% crystal violet in 20% methanol for 15 min. Colonies larger than 0.1 mm diameter were scored. The experiment was performed in triplicate for each cell line.

### Apoptosis assay

The apoptosis assay was conducted using an Annexin V-FITC/PI Apoptosis Detection Kit (BD Pharmingen, USA) following the manufacturer's protocol; assays were repeated three times. The results were analyzed using Cell Quest and flow cytometry (Beckman Coulter, USA) was used to distinguish the cells as viable (Annexin V-/PI-), early apoptotic (Annexin V+/PI-) or late apoptotic (Annexin V+/PI+).

### Wound healing and invasion assays

Cell migration was assessed by a scratch wound-healing assay. Cells were cultured in 6-well plate. After the cells reached sub-confluence, a scratching wound was generated with a sterile micropipette tip and the culture medium was replaced by serum-free DMEM, and the spread of wound closure was observed after 24 h and photographed under a microscope. Images were later analyzed by determining the distance between the cells on either side of the scratch overtime, and are represented in the figure as percent scratch closure.

For invasion assays, 5 × 10^4^ cells were seeded in a Matrigel-coated chamber (BD Biosciences) with 8 μm porosity present in the insert of a 24-well culture plate. FBS was added to the lower chamber as a chemo-attractant. After 16 h, the non-invading cells were gently removed with a cotton swab. Invasive cells located on the lower side of the chamber were fixed with 100% methanol for 20 min, stained with crystal violet for 15 min. Five random fields per well were taken, and cells were counted under a microscope. To test the effect of AKT dephosphorylation on the cell invasive abilities induced by TRIM29 expression, cells were pretreated with 20 μM AKT inhibitor VIII (MERCK) or 20 ng/ml of Rapamycin (Selleck Chemicals, USA) for 30 min before performing the invasion assays. Experiments were performed in triplicate.

RETRACTED

### Animal study

Six-week-old male athymic nude mice were injected subcutaneously with 4 × 10^6^ S18-TRIM29 or S18-control cells separately. The resulting tumors were examined every 3 days. Tumor size was measured using calipers, and tumor volumes were calculated (V = 0.5 × L × W^2^). After 40 days, the mice were sacrificed and the subcutaneous tumors were resected, fixed in 10% formalin, and embedded in paraffin blocks for hematoxylin-eosin (H&E) staining and IHC assay.

For the *in vivo* metastasis assays, 1 × 10^6^ S18 cells, stably expressing TRIM29 or the vector control, were injected intravenously through tail vein into each nude mice. The experiment was terminated after 8 weeks, the mice were examined and the liver and the lungs were removed and fixed with 10% formalin. Subsequently, consecutive tissue sections were made for each block of the liver and the lung, and stained with H&E. Finally, the numbers of the metastatic nodules were carefully examined and counted under microscope.

Animals were housed under standard conditions and cared for according to the institutional guidelines for animal care. The experiments were performed in accordance with the guidelines of the laboratory animal ethics committee of Sun Yat-sen University.

### Luciferase reporter assay

Oligonucleotides containing the wild-type (WT) or mutant (MT) puptative miR-335-5p or miR-15b-5p binding sites of the 3′-untranslated regions (3′-UTR) of the TRIM29 mRNA were ligated into the pMIR-REPORT vector (Ambion, Carlsbad, CA), respectively. 4×10^4^ cells per well were seeded in 24-well plates in triplicate. 24 h later, 100 ng firefly luciferase construct was co-transfected with 10 ng pRL-TK renilla plasmid into cells using Lipofectamine 2000 reagent (Invitrogen) in the presence of microRNA mimics, microRNA inhibitor or corresponding negative control. Media were replaced at 6 h, and the luciferase and renilla signals were measured 48 h after transfection using the Dual Luciferase Reporter Assay Kit (Promega), according to the manufacturer's protocol. The experiments were performed independently in triplicate.

### Statistical analysis

The Chi-square test was used for correlation analysis between clinicopathological features of patients with NPC and TRIM29 expression profiles. The linear correlations between TRIM29, p4E-BP1 and PTEN expression in NPC tissues were evaluated with Pearson correlation coefficient analysis. The Student's *t*-test (two-tailed) was used to evaluate significant differences between pairs of experimental data where appropriate. SPSS version 16.0 statistical software package was used for statistical analyses. *P* < 0.05 was regarded statistically significant (*P < 0.05; **P < 0.01; ***P < 0.001).

RETRACTED

## SUPPLEMENTARY MATERIAL TABLES



## References

[1] Cao SM, Simons MJ, Qian CN (2011). The prevalence and prevention of nasopharyngeal carcinoma in China. Chin J Cancer.

[2] Wee JT, Ha TC, Loong SL, Qian CN (2010). Is nasopharyngeal cancer really a “Cantonese cancer”?. Chin J Cancer.

[3] Lai SZ, Li WF, Chen L, Luo W, Chen YY, Liu LZ, Sun Y, Lin AH, Liu MZ, Ma J (2011). How does intensity-modulated radiotherapy versus conventional two-dimensional radiotherapy influence the treatment results in nasopharyngeal carcinoma patients?. Int J Radiat Oncol Biol Phys.

[4] Chua ML, Wee JT, Hui EP, Chan AT (2015). Nasopharyngeal carcinoma. Lancet.

[5] Jia WH, Huang QH, Liao J, Ye W, Shugart YY, Liu Q, Chen LZ, Li YH, Lin X, Wen FL, Adami HO, Zeng Y, Zeng YX (2006). Trends in incidence and mortality of nasopharyngeal carcinoma over a 20-25 year period (1978/1983-2002) in Sihui and Cangwu counties in southern China. BMC Cancer.

[6] Colaco RJ, Betts G, Donne A, Swindell R, Yap BK, Sykes AJ, Slevin NJ, Homer JJ, Lee LW (2013). Nasopharyngeal carcinoma: a retrospective review of demographics, treatment and patient outcome in a single centre. Clin Oncol (R Coll Radiol).

[7] Kapp LN, Painter RB, Yu LC, van Loon N, Richard CW, James MR, Cox DR, Murnane JP (1992). Cloning of a candidate gene for ataxia-telangiectasia group D. Am J Hum Genet.

[8] Borden KL (1998). RING fingers and B-boxes: zinc-binding proteinprotein interaction domains, Biochem. Cell Biol.

[9] Reddy BA, Etkin LD, Freemont PS (1992). A novel zinc finger coiled-coil domain in a family of nuclear proteins. Trends Biochem Sci.

[10] Reymond A, Meroni G, Fantozzi A, Merla G, Cairo S, Luzi L, Riganelli D, Zanaria E, Messali S, Cainarca S, Guffanti A, Minucci S, Pelicci PG, Ballabio A (2001). The tripartite motif family identifies cell compartments. EMBO J.

[11] Nisole S, Stoye JP, Saib A (2005). TRIM family proteins: retroviral restriction and antiviral defence. Nat Rev Microbiol.

[12] Wolf D, Goff SP (2007). TRIM28 mediates primer binding site-targeted silencing of murine leukemia virus in embryonic cells. Cell.

[13] Wang L, Heidt DG, Lee CJ, Yang H, Logsdon CD, Zhang L, Fearon ER, Ljungman M, Simeone DM (2009). Oncogenic function of ATDC in pancreatic cancer through Wnt pathway activation and beta-catenin stabilization. Cancer Cell.

[14] Hawthorn L, Stein L, Panzarella J, Loewen GM, Baumann H (2006). Characterization of cell-type specific profiles in tissues and isolated cells from squamous cell carcinomas of the lung. Lung Cancer.

RETRACTED

[15] Dyrskjøt L, Kruhøffer M, Thykjaer T, Marcussen N, Jensen JL, Møller K, Ørntoft TF (2004). Gene expression in the urinary bladder: a common carcinoma in situ gene expression signature exists disregarding histopathological classification. Cancer Res.

[16] Glebov OK, Rodriguez LM, Soballe P, DeNobile J, Cliatt J, Nakahara K, Kirsch IR (2006). Gene expression patterns distinguish colonoscopically isolated human aberrant crypt foci from normal colonic mucosa. Cancer Epidemiol Biomarkers Prev.

[17] Santin AD, Zhan F, Bellone S, Palmieri M, Cane S, Bignotti E, Anfossi S, Gokden M, Dunn D, Roman JJ, O'Brien TJ, Tian E, Cannon MJ, Shaughnessy J, Pecorelli S (2004). Gene expression profiles in primary ovarian serous papillary tumors and normal ovarian epithelium: identification of candidate molecular markers for ovarian cancer diagnosis and therapy. Int J Cancer.

[18] Mutter GL, Baak JP, Fitzgerald JT, Gray R, Neuberg D, Kust GA, Gentleman R, Gullans SR, Wei LJ, Wilcox M (2001). Global expression changes of constitutive and hormonally regulated genes during endometrial neoplastic transformation. Gynecol Oncol.

[19] Zhan F, Hardin J, Kordsmeier B, Bumm K, Zheng M, Tian E, Sanderson R, Yang Y, Wilson C, Zangari M, Anaissie E, Morris C, Muwalla F, van Rhee F, Fassas A, Crowley J, Tricot G, Barlogie B, Shaughnessy J (2002). Global gene expression profiling of multiple myeloma, monoclonal gammopathy of undetermined significance, and normal bone marrow plasma cells. Blood.

[20] Kosaka Y, Inoue H, Ohmachi T, Yokoe T, Matsumoto T, Mimori K, Tanaka F, Watanabe M, Mori M (2007). Tripartite motif-containing 29 (TRIM29) is a novel marker for lymph node metastasis in gastric cancer. Ann Surg Oncol.

[21] Schlomm T, Luebke AM, Sültmann H, Hellwinkel OJ, Sauer U, Poustka A, David KA, Chun FK, Haese A, Graefen M, Erbersdobler A, Huland H (2005). Extraction and processing of high quality RNA from impalpable and macroscopically invisible prostate cancer for microarray gene expression analysis. Int J Oncol.

[22] Ernst T, Hergenhahn M, Kenzelmann M, Cohen CD, Bonrouhi M, Weninger A, Klären R, Gröne EF, Wiesel M, Güdemann C, Küster J, Schott W, Staehler G, Kretzler M, Hollstein M, Gröne HJ (2002). Decrease and gain of gene expression are equally discriminatory markers for prostate carcinoma: a gene expression analysis on total and microdissected prostate tissue. Am J Pathol.

[23] Liu J, Welm B, Boucher KM, Ebbert MT, Bernard PS (2012). TRIM29 functions as a tumor suppressor in nontumorigenic breast cells and invasive ER+ breast cancer. Am J Pathol.

RETRACTED

[24] Zhang P, Zhang Z, Zhou X, Qiu W, Chen F, Chen W (2006). Identification of genes associated with cisplatin resistance in human oral squamous cell carcinoma cell line. BMC Cancer.

[25] Nacht M, Ferguson AT, Zhang W, Petroziello JM, Cook BP, Gao YH, Maguire S, Riley D, Coppola G, Landes GM, Madden SL, Sukumar S (1999). Combining serial analysis of gene expression and array technologies to identify genes differentially expressed in breast cancer. Cancer Res.

[26] Blanco-Aparicio C, Renner O, Leal JF, Carnero A (2007). PTEN, more than the AKT pathway. Carcinogenesis.

[27] Hill R, Wu H (2009). PTEN, stem cells, and cancer stem cells. J Biol Chem.

[28] Song LB, Li J, Liao WT, Feng Y, Yu CP, Hu LJ, Kong QL, Xu LH, Zhang X, Liu WL, Li MZ, Zhang L, Kang TB, Fu LW, Huang WL, Xia YF, Tsao SW, Li M, Band V, Band H, Shi QH, Zeng YX, Zeng MS (2009). The polycomb group protein Bmi-1 represses the tumor suppressor PTEN and induces epithelial-mesenchymal transition in human nasopharyngeal epithelial cells. J Clin Invest.

[29] Hosoi Y, Kapp LN, Murnane JP, Matsumoto Y, Enomoto A, Ono T, Miyagawa K (2006). Suppression of anchorage-independent growth by expression of the ataxia-telangiectasia group D complementing gene, ATDC. Biochem Biophys Res Commun.

[30] Ai L, Kim WJ, Alpay M, Tang M, Pardo CE, Hatakeyama S, May WS, Kladde MP, Heldermon CD, Siegel EM, Brown KD (2014). TRIM29 suppresses TWIST1 and invasive breast cancer behavior. Cancer Res.

[31] Avraham A, Cho SS, Uhlmann R, Polak ML, Sandbank J, Karni T, Pappo I, Halperin R, Vaknin Z, Sella A, Sukumar S, Evron E (2014). Tissue specific DNA methylation in normal human breast epithelium and in breast cancer. PLoS One.

[32] Sho T, Tsukiyama T, Sato T, Kondo T, Cheng J, Saku T, Asaka M, Hatakeyama S (2011). TRIM29 negatively regulates p53 via inhibition of Tip60. Biochim Biophys Acta.

[33] Tang ZP, Dong QZ, Cui QZ, Papavassiliou P, Wang ED, Wang EH (2013). Ataxia-telangiectasia group D complementing gene (ATDC) promotes lung cancer cell proliferation by activating NF-κB pathway. PLoS One.

[34] Liu Y, Chen LH, Yuan YW, Li QS, Sun AM, Guan J (2012). Activation of AKT is associated with metastasis of nasopharyngeal carcinoma. Tumour Biol.

[35] Tokunaga E, Oki E, Egashira A, Sadanaga N, Morita M, Kakeji Y, Maehara Y (2008). Deregulation of the Akt pathway in human cancer. Current cancer drug targets.

[36] Kalinsky K, Heguy A, Bhanot UK, Patil S, Moynahan ME (2011). PIK3CA mutations rarely demonstrate genotypic intratu- moral heterogeneity and are selected for in breast cancer progression. Breast cancer research and treatment.

[37] Whitehall VL, Rickman C, Bond CE, Ramsnes I, Greco SA, Umapathy A, McKeone D, Faleiro RJ, Buttenshaw RL, Worthley DL, Nayler S, Zhao ZZ, Montgomery GW, Mallitt KA, Jass JR, Matsubara N, Notohara K, Ishii T, Leggett BA (2012). Oncogenic PIK3CA mutations in colorectal cancers and polyps. Int J Cancer.

RETRACTED

[38] Li J, Yen C, Liaw D, Podsypanina K, Bose S, Wang SI, Puc J, Miliaresis C, Rodgers L, McCombie R, Bigner SH, Giovanella BC, Ittmann M, Tycko B, Hibshoosh H, Wigler MH, Parsons R (1997). PTEN, a putative protein tyrosine phosphatase gene mutated in human brain, breast, and prostate cancer. Science.

[39] Liotta LA (1986). Tumor invasion and metastases - role of the extracellular matrix: Rhoads Memorial Award lecture. Cancer Res.

[40] Wang W, Wen Q, Xu L, Xie G, Li J, Luo J, Chu S, Shi L, Huang D, Li J, Fan S (2014). Activation of Akt/mTOR pathway is associated with poor prognosis of nasopharyngeal carcinoma. PLoS One.

[41] Cai L, Ye Y, Jiang Q, Chen Y, Lyu X, Li J, Wang S, Liu T, Cai H, Yao K, Li JL, Li X (2015). Epstein-Barr virus-encoded microRNA BART1 induces tumour metastasis by regulating PTEN-dependent pathways in nasopharyngeal carcinoma. Nat Commun.

[42] Zhang LY, Ho-Fun Lee V, Wong AM, Kwong DL, Zhu YH, Dong SS, Kong KL, Chen J, Tsao SW, Guan XY, Fu L (2013). MicroRNA-144 promotes cell proliferation, migration and invasion in nasopharyngeal carcinoma through repression of PTEN. Carcinogenesis.

[43] Chen Q, Samaranayake LP, Zhou H, Xiao L (2000). Homozygous deletion of the PTEN tumor-suppressor gene is not a feature in oral squamous cell carcinoma. Oral Oncol.

[44] Schagdarsurengin U, Gimm O, Dralle H, Hoang-Vu C, Dammann R (2006). CpG island methylation of tumor-related promoters occurs preferentially in undifferentiated carcinoma. Thyroid.

[45] Bai W, Li W, Chen X, Wang T (2006). The relationship between hypermethylation of the PTEN promoter and laryngeal squamous cell carcinoma. Lin Chuang Er Bi Yan Hou Ke Za Zhi.

[46] Zhao YY, Tian Y, Zhang J, Xu F, Yang YP, Huang Y, Zhao HY, Zhang JW, Xue C, Lam MH, Yan L, Hu ZH, Dinglin XX, Zhang L (2014). Effects of an oral allosteric AKT inhibitor (MK-2206) on human nasopharyngeal cancer in vitro and in vivo. Drug Des Devel Ther.

[47] Qin J, Ji J, Deng R, Tang J, Yang F, Feng GK, Chen WD, Wu XQ, Qian XJ, Ding K, Zhu XF (2015). DC120, a novel AKT inhibitor, preferentially suppresses nasopharyngeal carcinoma cancer stem-like cells by downregulating Sox2. Oncotarget.

[48] Liu T, Sun Q, Li Q, Yang H, Zhang Y, Wang R, Lin X, Xiao D, Yuan Y, Chen L, Wang W (2015). Dual PI3K/mTOR inhibitors, GSK2126458 and PKI-587, suppress tumor progression and increase radiosensitivity in nasopharyngeal carcinoma. Mol Cancer Ther.

